This article has been retracted.

# Fluoride Exposure Suppresses Proliferation and Enhances Endoplasmic Reticulum Stress and Apoptosis Pathways in Hepatocytes by Downregulating Sirtuin-1

**DOI:** 10.1155/2022/7380324

**Published:** 2022-08-21

**Authors:** Yanlong Yu, Ling Li, Wenfeng Yu, Zhizhong Guan

**Affiliations:** ^1^Key Laboratory of Endemic and Ethnic Diseases, Ministry of Education, Guizhou Medical University, Guiyang, China; ^2^School of Basic Medical Science, Guizhou Medical University, Guiyang 550002, China

## Abstract

**Objective:**

To explore the function and mechanism of Sirt-1 in fluorine-induced liver injury.

**Method:**

Fluorosis rats were first established. The fluorine content, pathological structure, collagen fibers, and fibrosis in liver tissues were tested through the fluoride ion selective electrode method, H&E, Masson, and Sirius red staining; alanine aminotransferase (ALT), aspartate aminotransferase (AST), interleukin 18 (IL-18), and tumor necrosis factor-*α* (TNF-*α*) levels in rat serum were also analyzed using ELISA kits. Then, the fluorosis cell model was built, which was also alleviated with NaF, Sirt-1 siRNAs, or endoplasmic reticulum stress (ERS) alleviator (4-PBA). CCK-8 also assessed cell proliferation; RT-qPCR or Western blots detect sirtuin-1 (Sirt-1), protein kinase R- (PKR-) like endoplasmic reticulum kinase (PERK), and endoplasmic reticulum stress (ERS) and apoptosis-related protein levels in liver tissue.

**Results:**

Our results uncovered that fluorine exposure could aggravate the pathological damage and fibrosis of rat liver tissues and increase indicators related to liver injury. And fluoride exposure also could downregulate Sirt-1 and upregulate ERS-related proteins (PERK, 78-kD glucose-regulated protein (GRP-78), and activating transcription factor 6 (ATF6)) and apoptosis-related protein (caspase-3 and C/EBP-homologous protein (CHOP)) in rat liver tissues. Besides, we proved that fluoride exposure could suppress proliferation and enhances ERS and apoptotic pathways in AML12 cells by downregulating Sirt-1. Moreover, we revealed that ERS alleviator (4-PBA) could induce proliferation and prevent ERS and apoptosis in fluorine-exposed AML12 cells.

**Conclusions:**

We suggested that fluorine exposure can induce hepatocyte ERS and apoptosis through downregulation of Sirt-1.

## 1. Introduction

Fluorine exists in the environment in the form of fluoride [1]. And fluorine is a vital trace element present in humans and animals, mainly in bones and teeth [2, 3]. While long-term exposure to fluoride in the air, food, and water can lead to fluorosis, it can also cause dental fluorosis and fluorosis bone disease [4]. It has also been confirmed that chronic fluorosis can result in extensive pathological damage to the body [5]. Excessive intake of fluorine will cause morphological, functional, and metabolic changes in various organs, exposing soft tissues such as the liver, nerves, kidneys, blood vessels, and muscles to fluorine damage [6, 7]. The liver is the largest tissue organ in the body and can be involved in metabolism and blood production. Besides, the liver is the main organ for removing toxic substances from living organisms [8]. Long-term chronic fluoride exposure can lead to the accumulation of large amounts of fluoride in the liver, destroying its tissue morphology and affecting its normal physiological functions [9]. Several studies have indicated that sodium fluoride (NaF) can induce mitochondrial damage and promote hepatotoxicity and cellular damage [10, 11]. However, the mechanism of NaF-induced hepatotoxicity has not been clearly elucidated.

The endoplasmic reticulum (ER) is the site of protein synthesis, folding, and quality control [12]. During stressful conditions, unfolded and misfolded proteins can accumulate in the ER lumen, eventually causing ER stress (ERS) [13]. Research showed that ERS is associated with liver injury, and ERS-associated apoptosis is present throughout the process of liver injury [14]. Therefore, regulating ERS-associated apoptosis is very important to prevent liver injury.

Histone deacetylase (HDAC) can modify chromatin structure and regulate transcription factor activity [15]. And sirtuin-1 (Sirt-1) is a class III HDAC and can regulate biological processes including cellular metabolism, gene transcription, immune response, and glucose homeostasis through multiple deacetylation factors [16]. Sirt-1 has been reported to be associated with cell growth, apoptosis, senescence, autophagy, and other activities, which plays a key role in several diseases, such as neurodegenerative diseases, metabolic diseases, and cancer [17–19]. Several researchers have also confirmed that Sirt-1 is relevant to liver injury [20–22]. Besides, Sirt-1 also can exert a protective role against liver injury by suppressing ERS [23]. Recent study also revealed that Sirt-1 can weaken ERS by inhibiting the protein kinase R- (PKR-) like endoplasmic reticulum kinase- (PERK-) eIF2*α*-activating transcription factor 4 (ATF4) pathway, ultimately reducing ERS-induced apoptosis [24]. However, whether Sirt-1 can be involved in fluorine exposure-induced ERS in hepatocytes is not fully understood.

## 2. Materials and Methods

### 2.1. Animal

Twenty-four healthy Wistar rats (males, 8 weeks old) were purchased from Guizhou Medical University. Animal Center provided with a standard diet as well. All animals were kept under standard laboratory conditions: 18-22°C, good ventilation, certain humidity, sanitary conditions, and free access to water and food. After 1 week of acclimatization, the rats were randomly divided into 3 groups (8 animals per group), which were given deionized water containing 0, 10, and 50 mg/L sodium fluoride (NaF). After 8 weeks, blood was collected from the eyes, and serum was obtained by centrifugation based on the animal ethical standards. After cardiac perfusion, the livers were preserved in 10% formalin for histological examination. The remaining liver samples were placed in liquid nitrogen. Animals were conducted in the light of the standard regulations and guidelines, and the Experimental Animal Ethics Committee approved the experiments of Guizhou Medical University (No. 2103001).

### 2.2. Cell Culture

Alpha mouse liver 12 (AML12, CRL-2254) cells were from ATCC. And AML12 cells were grown in DMEM/F12 (Gibco, USA) with 1% insulin-transferrin-selenium (ITS; Gibco, 41400045), 10% fetal bovine serum (FBS, Gibco), and 40 ng/mL dexamethasone at 37°C, 5% CO_2_.

### 2.3. Cell Processing

AML12 cells were processed with 0, 10, 25, 50, 75, and 100 mg/L NaF for 36 h, respectively. Besides, AML12 cells were treated with 50 mg/L NaF and 1 mM 4-PBA. Sirt-1 siRNAs and negative control (NC) were from GenePharma (Suzhou, China). Then AML12 cells (density about 60%) in a 6-well plate were dealt with 50 mg/L NaF and transfected with 50 nM Sirt-1 siRNAs and 50 nM NC using Lipofectamine 3000 (Invitrogen) following the instructions.

### 2.4. Fluoride Ion Selective Electrode Method

Working curve preparation: 0, 1.0, 2.0, 3.0, 4.0, and 5.0 *μ*g of fluorine standard solution was placed in a 50 mL volumetric flask. 1.00 g of liver tissue was ground into powder, filtered, and placed in a 50 mL volumetric flask. Each volumetric flask was added with 10 mL of hydrochloric acid, soaked airtight for 1 h, and added with 25 mL of total ionic strength buffer. After connecting to the measuring instrument, the electrode was inserted into a 25 mL plastic cup filled with water. After the potential value was balanced, the potential of the standard solution and the sample solution was measured, respectively.

### 2.5. H&E Staining

Based on the research reported [25], at the end of the experiment, all rats were decollated to death, and liver tissues were taken. The liver tissues were fixed in 4% neutral formaldehyde for 48 h, dehydrated in ethanol gradient, and embedded in paraffin wax to produce pathological sections of 3 *μ*m thickness. After washing, the sections were dyed with Harris hematoxylin for 5 min, 1% hydrochloric acid alcohol, and 0.6% ammonia returned to blue. Then, the sections were colored with Eosin for 1 min, dehydrated, and processed with xylene. After sealing with neutral gum, the pathologic structure was confirmed with a light microscope.

### 2.6. Masson Staining

Based on the research reported [26], after conventional dewaxing, the sections were stained with hematoxylin for 10 min, rinsed with running water for 1 min, placed in static water for 5 min, dyed with Ponceau staining solution for 7 min, washed with 2% glacial acetic acid for 5 s, fractionated with 1% phosphomolybdic acid for 10 min, colored with aniline blue for 5 min, and washed with 2% glacial acetic acid for 5 s. The results were examined under a microscope.

### 2.7. Sirius Red Staining

Based on the research reported [27], after conventional dewaxing, the sections were stained with Harris hematoxylin for 5 min and Sirius red dye for 20 min. After dehydration and transparency, the sections were photographed under a microscope.

### 2.8. ELISA

Based on the instructions and research report [28], the levels of alanine aminotransferase (ALT), aspartate aminotransferase (AST), interleukin 18 (IL-18), and tumor necrosis factor-*α* (TNF-*α*) in rat serum were analyzed using the respective ELISA kits. The kits included ALT ELISA Kit (Nanjing Jiancheng Bioengineering Institute, China), AST ELISA Kit (Abcam, Cambridge, UK), IL-18 ELISA Kit (Elabscience Biotechnology, China, E-EL-M0730c), and TNF-*α* ELISA Kit (Multi-Science Co. Ltd., Hangzhou, China, EK282/3-24).

### 2.9. RT-qPCR Assay

Based on the research reported [29], approximately 100 mg of rat liver tissue from each group was repeatedly ground, and AML12 cells from each group were collected separately. Total RNAs were isolated from the samples with TRIzol (TAKARA; cat. no. 9109). Based on the kit instructions, reverse transcription was conducted using BestarTM qPCR RT kit (DBI, cat. no. 2220). And Sirt-1 and PERK expressions were tested with BestarTM qPCR MasterMix (DBI, cat. no. 2043). And the data was counted with the 2^-△△Ct^ method. The primers used for the qPCR analysis in this study are listed in Table 1.

### 2.10. Western Blot Assay

Based on the research reported [30], the samples in each group were supplemented with 1 mL of RIPA buffer with protease inhibitor (Sigma, USA). Supernatant (total protein) was collected after high-speed centrifugation. After quantification with the BCA method, 30 *μ*g protein was added to the loading buffer for denaturation. Each group of total proteins was subjected to SDS-PAGE electrophoresis, and the proteins were transferred to the PVDF membrane (Millipore). Protein was incubated overnight at 4°C with primary antibody (Abcam, Cambridge, MA, USA) and then incubated for 1 h at room temperature with HRP-coupled secondary antibody (Abcam). After TBST cleaning, ECL chemiluminescence substrate (Pierce, #32106) was applied for color rendering.

### 2.11. CCK-8 Assay

Based on the research reported [31], AML12 cells were collected, resuspended, and counted. 100 *μ*L of AML12 cells (2 × 10^3^) in a complete medium was inoculated in 96-well plates and processed in line with the experimental objectives. After incubation at 37°C for 0, 12, 24, and 36 h, each well was replaced with a medium containing 10% CCK-8 (Dojindo, Rockville, MD, USA) for 2 h. The absorbance of each group was tested at 450 nm on a microplate.

### 2.12. Statistical Analysis

The experiments were independently replicated 3 times. All data were presented as mean ± SD and analyzed using SPSS 20.0 software (SPSS, Inc., Chicago, IL, USA). When the variance of the data was consistent, data were compared using a one-way analysis of variance (ANOVA). *P* < 0.05 was also regarded as statistically significant.

## 3. Results

### 3.1. Fluorine Exposure Induces Liver Injury and Liver Fibrosis in Rats

To investigate the impact of fluorine exposure on the pathological structure of rat liver tissues, we fed rats with 10 and 50 mg/L NaF. After 8 weeks, we found that relative to the control group, the amount of fluorine in liver tissues was dramatically raised in the fluorine-treated group, especially the 50 mg/L NaF group (Figure 1(a)). In this way, we determined that fluorine was markedly elevated in the liver tissue of NaF-treated rats. Then, we collected liver tissues from each group. H&E staining results signified that normal drinking rats had normal morphology of hepatocytes with neat arrangement and no pathological changes in the liver tissue structure. NaF-fed rats showed obvious inflammatory cell infiltration in the liver tissues with disorganized cell arrangement and pathological changes. Histopathological changes in the liver tissues were significantly higher in the 50 mg/L NAF group than in the 10 mg/L NAF group (Figure 1(b)). Then, Masson staining data denoted that the collagen fibers were observably increased in NAF treatment groups relative to that in the control, especially the 50 mg/L NAF group (Figure 1(c)). Meanwhile, Sirius-red staining showed that after 8 weeks of NAF treatment, fibrosis in rat liver tissues was signally aggrandized compared with the control group. The 50 mg/L NAF group was higher than the 10 mg/L NAF group (Figure 1(d)). Moreover, we proved that the levels of ALT, AST, IL-18, and TNF-*α* in rat serum were notably higher in the NAF-treated groups than in the control group, especially in the 50 mg/L NAF group (Figure 1(e)). With these data, we demonstrated that fluorine exposure has a remarkable induction effect on liver injury and fibrosis in rats.

### 3.2. Effects of Fluoride Exposure on Sirt-1, ERS, and Apoptosis Pathways in Rats

Next, we verified the possible mechanism of fluoride exposure affecting liver injury and fibrosis. By RT-qPCR, we found that fluoride exposure (especially 50 mg/L NAF) could memorably downregulate Sirt-1 in rat liver tissues, revealing that Sirt-1 may be a potential regulator gene of fluoride exposure-induced liver injury (Figure 2(a)). Meanwhile, we proved that NAF administration could prominently upregulate PERK in rat liver tissues, and 50 mg/L NAF has a stronger regulatory effect than 10 mg/L NAF (Figure 2(b)). PERK is a transmembrane protein kinase on the endoplasmic reticulum membrane associated with ERS [32]. In this way, we hypothesize that the effect of fluoride exposure on liver injury may be related to ERS. And then, Western blot data displayed that fluoride exposure (especially 50 mg/L NAF) could decrease Sirt-1 expression and increase expressions of ERS-related proteins, including PERK, GRP-78, and ATF6, and apoptosis-related proteins, including caspase-3 and CHOP in liver tissues (Figures 2(c) and 2(d)). Overall, we testified that fluoride exposure could downregulate Sirt-1 and induce ERS and apoptosis pathways in rats.

### 3.3. Fluoride Exposure Suppresses Proliferation, Downregulates Sirt-1, and Enhances ERS and Apoptotic Pathways in AML12 Cells

Based on the function and mechanism of fluoride exposure in rats, we further analyzed the role of fluoride exposure in cells in vitro. We first cultured the AML12 cells and treated them for 36 h with 0, 10, 25, 50, 75, and 100 mg/L NaF. CCK-8 results denoted that NaF administration could observably suppress AML12 cell proliferation, and the higher the concentration of NaF, the lower the cell proliferation capacity (Figure 3(a)). Besides, RT-qPCR data represented that fluoride exposure (10 and 50 mg/L NaF) could memorably upregulate PERK and downregulate Sirt-1 in AML12 cells (Figures 3(b) and 3(c)). And Western blot results also manifested that NaF treatment could cause prominent increases in PERK, GRP-78, ATF6, CHOP, and caspase-3 protein expressions and a noteworthy decrease of the Sirt-1 protein expression in AML12 cells (Figures 3(d) and 3(e)). So, this part of the data revealed that fluoride exposure also could result in proliferation inhibition and ERS and apoptosis induction in AML12 cells.

### 3.4. Sirt-1 Knockdown Enhances Suppression of Proliferation and Induction of ERS and Apoptosis Mediated by Fluorine Exposure in AML12 Cells

As we demonstrated, fluoride exposure could downregulate Sirt-1 in liver tissues and AML12 cells, suggesting a critical role for Sirt-1 in liver injury. And we further explored whether Sirt-1 silencing can affect AML12 cell proliferation, ERS, and apoptosis mediated by fluorine exposure. 50 mg/L NaF and 50 nM Sirt-1 siRNAs were applied to treat or transfect AML12 cells. We first uncovered that the decrease in the Sirt-1 expression mediated by fluorine exposure could be further enhanced by Sirt-1 silencing in AML12 cells (Figure 4(a)). And CCK-8 results signified that Sirt-1 knockdown also could further enhance the diminished proliferative capacity induced by fluoride exposure in AML12 cells (Figure 4(b)). We also disclosed that Sirt-1 knockdown could further amplify the elevated PERK, GRP-78, ATF6, CHOP, and caspase-3 expressions and reduced the Sirt-1 expression mediated by fluoride exposure in AML12 cells (Figures 4(c) and 4(d)). Thus, we certified that Sirt-1 knockdown could further induce the effects of fluorine exposure on AML12 cell proliferation, ERS, and apoptosis.

### 3.5. ERS Alleviator (4-PBA) Induces Proliferation and Weakens ERS and Apoptosis in Fluorine-Exposed AML12 Cells

On account of the above data, fluorine exposure can induce ERS of AML12 cells by downregulating Sirt-1. We further determined the influence of ERS alleviator (4-PBA) on proliferation, ERS, and apoptosis in fluorine-exposed AML12 cells. We first discovered that the reduction in AML12 cell proliferation capacity induced by fluorine exposure was partially reversed after 4-PBA processing (Figure 5(a)). And our data also exhibited that 4-PBA treatment could partly weaken the fluorine exposure-mediated downregulation of Sirt-1 and upregulations of ERS-related proteins (PERK, GRP-78, and ATF6) and apoptosis-related protein (caspase-3 and CHOP)) in AML12 cells (Figures 5(b) and 5(c)). Overall, we verified that the diminished proliferation and enhanced ERS and apoptosis mediated by fluorine exposure could be reversed by ERS alleviator (4-PBA) in AML12 cells.

## 4. Discussion

Fluoride is widely present in the natural environment [33]. And long-term fluorine exposure can have certain toxic effects on the organism and cause significant hepatic pathological damage [34]. Currently, a study demonstrated that fluoride exposure could cause liver damage by the mitochondrial apoptosis pathway [9]. AST and ALT are the earliest and most sensitive indicators of the appearance of liver injury [35]. When liver tissue is necrotic or damaged, ALT and AST escape from hepatocytes and enter the bloodstream, significantly increasing serum ALT and AST activity [36]. Therefore, the increase of ALT and AST activity in serum reflects the degree of hepatocellular injury to a certain extent. In our study, we further proved that NaF treatment could induce necrosis and nuclear sequestration in hepatocytes and reduce intracellular organelles and swollen mitochondria in liver tissues of rats. Meanwhile, NaF also could elevate the levels of liver injury-related indicators (ALT and AST) and inflammatory indicators (IL-18, TNF-*α*) in rat serum. These results suggested that fluorine could induce liver injury in a dose-dependent manner.

Hepatic fibrosis (HF) is a repair response of the liver in response to chronic injury [37]. HF is also an intermediate stage in the progression of chronic liver disease to cirrhosis, which is a key stage in reversing the disease [38]. Late-stage HF may progress to irreversible cirrhosis [39]. And cirrhosis may further cause ascites, splenomegaly, formation of collateral circulation, upper gastrointestinal bleeding, and even death [40]. Our data further verified that fluorine exposure also could accelerate liver fibrosis in rats. Therefore, fluorine exposure can enhance liver injury and induce liver fibrosis.

Fluorosis is mainly associated with oxidative stress, hormonal regulation, and apoptosis [41]. Research showed that signaling pathways and related factors are relevant to fluorosis [42, 43]. To further explore the underlying mechanisms of fluorosis-induced liver injury, we investigated the effects of fluorine on hepatocyte ERS and apoptotic pathways. Apoptosis, a form of programmed cell death, can be induced by different toxic stimuli [44]. The literature reported that excess NaF could cause apoptosis in different cell types, including osteoblasts and human embryonic stem cells [45, 46]. And ERS is one of the key pathways of fluorine-induced apoptosis [47]. ERS acts as a cellular self-protection mechanism and normally has a role in protecting cells from damage. Adverse environments, such as oxidative stress and toxic stimuli, can accumulate unfolded and misfolded proteins in the ER, which can activate the unfolded protein response (UPR) [48]. UPR can maintain the balance of ER quantity and normal function in the body during ERS. Under stress, GRP78 can activate ERS through PERK, ATF6, and IRE1 [49]. While excessive ERS instead can activate ERS-associated apoptotic proteins such as CHOP, it can eventually trigger apoptosis [50]. In vivo study also showed that high fluorine concentrations can induce ERS and apoptosis in osteoblasts [51]. Our study further verified that fluoride exposure could upregulate ERS-and apoptosis-related proteins in liver tissues and AML12 cells. Thus, fluoride exposure could induce ERS and apoptosis in hepatic cells. Meanwhile, we discovered that ERS alleviator (4-PBA) could induce proliferation and inhibit ERS and apoptosis in fluorine-exposed AML12 cells, suggesting that fluorine exposure to hepatocyte ERS is critical.

More importantly, our data showed that fluoride exposure could prominently downregulate Sirt-1 in liver tissues and AML12 cells. Sirt-1 is a deacetylase that can regulate biological metabolism through deacetylation [52]. Besides, Sirt-1 has been reported to play key regulatory roles in physiological processes such as apoptosis, differentiation, oxidative stress, senescence, signaling, transcriptional regulation, and metabolic regulation through the regulation of histones, NF-*κ*B, FOXO, and p53 [53, 54]. In recent years, studies confirmed that Sirt-1 is essential in liver-related diseases, such as liver transplantation [55], liver ischemia/reperfusion injury [56], liver fibrosis [57], fatty liver [58], alcoholic liver injury, and fibrosis [59]. At the same time, the role and mechanism of Sirt-1 in liver injury induced by fluoride exposure are unclear. Our results further indicated that Sirt-1 knockdown could further enhance the induction of ERS and apoptosis mediated by fluorine exposure in AML12 cells.

In our study, we first constructed fluorosis rat and cell models using NaF and clarified the influences of fluorine exposure on liver injury and fibrosis in rats. Besides, we explored the impacts of fluorine exposure on ERS- and apoptosis-related proteins in fluorosis rats and cells. Moreover, we further verified the action of Sirt-1 silencing and ERS alleviator (4-PBA) in fluorine-exposed rat liver tissues in vivo and AML12 cells in vitro. Therefore, the investigation of the protective mechanism of SIRT-1 against fluoride exposure-induced liver injury may provide a laboratory basis for the future clinical mitigation of fluorosis.

## 5. Conclusion

We demonstrated that fluorine exposure could induce hepatocyte injury through modulation of ERS and apoptotic pathways. Besides, Sirt-1 knockdown could further enhance the ERS and apoptotic processes in hepatocytes induced by fluoride exposure and enhance the toxic effects of NaF (Figure 6).

## Figures and Tables

**Figure 1:** Fluorine exposure induces liver injury and liver fibrosis in rats. The Wistar rats were fed with water containing 0, 10, and 50 mg/L sodium fluoride (NaF) for 8 weeks, respectively. (a) Fluorine content in liver tissues was monitored via fluoride ion selective electrode method. (b) Alterations in the pathological structure of the rat liver tissues were assessed through H&E staining, magnification, ×200. (c) The collagen fibers were tested by Masson staining in rat liver tissues, magnification, ×200. (d) Sirius red staining was adopted to analyze the fibrosis in rat liver tissues, magnification, ×200. (e) ELISA kits were utilized to evaluate the levels of ALT, AST, IL-18, and TNF-*α* in rat serum. ^∗∗∗^*P* < 0.001.

**Figure 2:** Effects of fluoride exposure on Sirt-1, ERS, and apoptosis pathways in rats. 10 and 50 mg/L NaF were applied to feed the Wistar rats. (a, b) RT-qPCR analysis of Sirt-1 and PERK expressions in liver tissues. (c) Western blot demonstrated the changes in PERK, Sirt-1, GRP-78, ATF6, CHOP, and caspase-3 expressions in liver tissues. (d) Quantitative analysis of the above Western blot results. ^∗∗^*P* < 0.01, ^∗∗∗^*P* < 0.001.

**Figure 3:** Fluoride exposure suppresses proliferation, downregulates Sirt-1, and enhances ERS and apoptotic pathways in AML12 cells. AML12 cells were first processed with 0, 10, 25, 50, 75, and 100 mg/L NaF for 36 h. (a) Cell proliferation was determined by CCK-8. (b, c) PERK and Sirt-1 expressions were assessed through RT-qPCR. (d) Western blot was adopted to confirm the protein expressions of PERK, Sirt-1, GRP-78, ATF6, CHOP, and caspase-3. (e) The above six proteins were quantified separately in line with grayscale values. ^∗^*P* < 0.05, ^∗∗^*P* < 0.01, ^∗∗∗^*P* < 0.001.

**Figure 4:** Sirt-1 knockdown enhances suppression of proliferation and induction of ERS and apoptosis mediated by fluorine exposure in AML12 cells. AML12 cells were addressed with 50 mg/L NaF and transfected with Sirt-1 siRNAs. (a) RT-qPCR exhibited the change in the Sirt-1 expression. (b) CCK-8 was utilized to confirm the change of cell proliferation. (c) Western blotting analysis of PERK, Sirt-1, GRP-78, ATF6, CHOP, and caspase-3 expressions in AML12 cells. (d) Individual proteins were quantified. ^∗^*P* < 0.05, ^∗∗∗^*P* < 0.001 vs. control group; ^&^*P* < 0.05, ^&&&^*P* < 0.001 vs. F50+ Sirt-1/Ko group. Ko: gene knockout.

**Figure 5:** ERS alleviator (4-PBA) induces proliferation and weakens ERS and apoptosis in fluorine-exposed AML12 cells. (a) CCK-8 presented the proliferation change in AML12 cells processed with NaF and 4-PBA. (b) PERK, Sirt-1, GRP-78, ATF6, CHOP, and caspase-3 expressions were credited by applying Western blot in AML12 cells after administration with NaF and 4-PBA. (c) The gray value of each protein was quantified, respectively. ^∗^*P* < 0.05, ^∗∗∗^*P* < 0.001 vs. control group; ^&^*P* < 0.05, ^&&&^*P* < 0.001 vs. F50 group.

**Figure 6:** Schematic representation of the process that SIRT-1 against fluoride exposure-induced liver injury.

**Table 1:** Primer sequences for RT-PCR.

Target gene	Primer	Primer sequences
Sirt-1	F	5′-ACGCTGGAACAGGTTGCGGG-3′
	R	5′-AGCGGTTCATCAGCTGGGCAC-3′
PERK	F	5′-GCTCAAAGACGAAAGCACAGAC-3′
	R	5′-CCCACCGAGAAAGACCGAC-3′
*GAPDH*	F	5′-ACCACAGTCCATGCCATCAC-3′
	R	5′-TCCACCACCCTGTTGCTGTA-3′

## Data Availability

The datasets used and/or analyzed during the current study are available from the corresponding authors on reasonable request.
